# Using an Optimized Learning Vector Quantization- (LVQ-) Based Neural Network in Accounting Fraud Recognition

This article has been retracted.

**DOI:** 10.1155/2021/4113237

**Published:** 2021-06-28

**Authors:** Yuan Zheng, Xiaolan Ye, Ting Wu

**Affiliations:** ^1^School of Finance, Anhui University of Finance and Economics, Bengbu, Anhui 233030, China; ^2^School of Insurance, Southwestern University of Finance and Economics, Chengdu, Sichuan 611130, China; ^3^School of Computer Science, ZhongYuan University of Technology, Zhengzhou, Henan 450007, China

## Abstract

With the continuous development and wide application of artificial intelligence technology, artificial neural network technology has begun to be used in the field of fraud identification. Among them, learning vector quantization (LVQ) neural network is the most widely used in the field of fraud identification, and the fraud identification rate is relatively high. In this context, this paper explores this neural network technology in depth, uses the same fraud sample to test the fraud recognition rate of these two models, and proposes an optimized LVQ-based combined neural network fraud risk recognition model on this basis. This paper selects 550 listed companies that have committed fraud from 2015 to 2019 as the fraud samples, determines 550 nonfraud matching sample companies in accordance with the Beasley principle one-to-one, and uses this as the research sample. The fraud risk identification indicators with better identification effects combed out according to the literature were used as the initial indicator system. After the collinearity problem was eliminated through the paired sample *T* test and principal component analysis, the five indicators with the best identification effects were finally selected. Finally, based on the above theoretical analysis and empirical research summarizing the full text, it analyzes the shortcomings of this research and puts forward prospects for the future development of fraud risk identification models.

## 1. Introduction

Fraud has severely affected the public's confidence in the accounting community and the capital market; how to effectively identify corporate fraud has become the top priority of accounting theory, practice, and regulatory agencies. The empirical research shows that the model fraud identification effect is better than the fraud case analysis, and the construction of an effective fraud risk identification model is inseparable from perfect fraud identification indicators and appropriate identification methods. At present, the research on fraud identification indicators has been relatively complete, but there is less research on fraud identification models. The concept of fraud does not have a unified conclusion. Governments or regulatory agencies at home and abroad have defined it. For example, the National Antifraud Accounting Reporting Committee (Treadway Committee) defines accounting fraud as “a deliberate or reckless act. Whether it is false reporting or omissions, the result is a major misleading accounting report.” In addition, scholars have also defined accounting fraud [1, 2]. Hormozzadefighalati defined accounting fraud as fraudulent use of accounting fraud and other violations or illegal means to seek self-interest, thereby harming the interests of others' intentional behavior [3]. Wang et al. believed that the accounting fraud company executives have deceptively manipulated accounting reports [4]. Siamidoudaran et al. put forward on the basis of summarizing and analyzing the existing literature: accounting fraud is the intention of the perpetrator to obtain illegitimate benefits, deliberately violate the principle of authenticity in a planned, purposeful, and targeted manner, and violate the state. Acts of laws, regulations, policies, and rules ultimately lead to distortion of accounting information [5]. Based on the above definition of accounting fraud, the definition of accounting fraud in this article is as follows: in order to seek illegitimate benefits, the management of a company deliberately uses forgery, tampering, cover-up, and other deceptive methods to deliberately cause the distortion of accounting information. The types of accounting fraud mainly include illegal purchase of stocks, false statements, violations of capital contributions, and violations of regulations Hype and so on.

Environment refers to all external things that surround a certain thing and have some influence on it; that is, environment refers to the surrounding things that are relative and related to a certain central thing. Any enterprise or social organization exists in the environment. The corporate environment refers to a collection of interrelated, mutually restrictive, and constantly changing factors that affect corporate management decisions and production and operation activities. The internal environment of an enterprise refers to the sum of the material and cultural environment within the enterprise. The external environment of an enterprise refers to the sum of the political environment, economic environment, social environment, and technological environment outside the enterprise. According to the definition of environment and corporate environment, this article believes that the environment of accounting fraud refers to a collection of interrelated, mutually restrictive, and constantly changing factors that affect the existence of accounting fraud, including internal environmental characteristics and external environmental characteristics. Because accounting fraud is carried out by the company as a carrier, the environmental characteristics of accounting fraud refer to the environment that affects accounting fraud inside and outside the company. The following article will introduce the internal and external environmental characteristics of accounting fraud.

The internal environmental characteristics of accounting fraud refer to the collection of various factors that exist within the enterprise and affect accounting fraud [6]. Specifically, it includes corporate governance structure, institutional settings, the implementation of the system, and so on. The internal environment of accounting fraud affects the size of the opportunity for company managers to commit fraud, the probability of fraud being discovered, and the nature and degree of punishment of fraudsters after fraud is discovered. A sound internal mechanism will greatly reduce the probability of accounting fraud, and there are loopholes where defective internal mechanism will increase the possibility of accounting fraud. In the research of Brinkrolf et al. [7], it contains two internal environmental characteristics of accounting fraud, the company's internal governance structure and the company's operating performance. The internal environmental characteristics of accounting fraud studied in this article include board structure, director encouragement, leadership structure, ownership structure, and executive incentives.

The external environmental characteristics of accounting fraud refer to the collection of various factors that exist outside the enterprise and affect accounting fraud. It specifically includes external corporate governance, market environment, political environment, and economic environment. The external environment of accounting fraud affects the chances of fraud by company managers, the probability of fraud being discovered, and the nature and degree of punishment of fraudsters after fraud is discovered. The supervision and governance of fraudsters by the external environment is a beneficial supplement to the internal environment. The market system, favorable political and economic environment, and effective supervision system can reduce the possibility of accounting fraud. On the contrary, if the market environment, political environment, and economic environment cannot effectively supervise accounting fraud, then the occurrence of accounting fraud possibility will increase. The external environment of accounting fraud studied in this article includes the quality of external auditing, the degree of media development, the degree of institutional and legal constraints, and the degree of product competition. With the continuous development and wide application of artificial intelligence technology, artificial neural network technology has begun to be used in the field of fraud identification. Among them, the LVQ neural network is the most widely used in the field of fraud identification, and the fraud identification rate is relatively high. In this context, this paper explores this neural network technology in depth, uses the same fraud sample to test the fraud recognition rate of these two models, and proposes an optimized LVQ-based combined neural network fraud risk recognition model on this basis. This paper selects listed companies that have committed fraud from 2015 to 2019 as the fraud samples, uses the fraud risk identification indicators with better identification results combed out according to the literature as the initial indicator system, and eliminates the commonality through paired sample *T* test and principal component analysis. After the linear problem, the 5 indicators with the best recognition effect were finally selected. Finally, based on the above theoretical analysis and empirical research summarizing the full text, it analyzes the deficiencies in this research and puts forward a prospect for the future development of the fraud risk identification model.

## 2. LVQ Neural Network

### 2.1. Concept and Structure of LVQ Neural Network Model

The LVQ neural network is proposed on the basis of the competitive network structure and belongs to the forward neural network. The LVQ neural network combines the idea of competitive learning with supervised learning algorithms [8]. In the process of network learning, the assignment category of input samples is specified through the tutor signal, thereby overcoming the lack of classification information caused by the use of unsupervised learning algorithms in self-organizing networks weakness. The biggest advantage of LVQ neural network is that it cannot only classify linear input data, but also process multidimensional data containing noise interference. LVQ neural network has a wide range of applications in the field of optimization and pattern recognition, and it is also one of the typical classification models. Similar to BP neural network, LVQ neural network also has three network layers, which are divided into input layer, competition layer, and linear layer. There is a complete connection between the input layer and the competition layer [9].

The competition layer classifies the learning of the input vector as the same as the competition layer and calls the classification of the competition layer as subcategories. There is a partial connection between the competition layer and the linear layer. The linear layer mainly maps the classification results of the competition layer to the target classification results according to the needs of users, and the classification of the linear layer is called the target classification. The specific LVQ neural network model structure and data processing process are shown in Figures 1 and 2:

The output of each neuron in the competition layer and the linear layer corresponds to a subclassification or target classification result, so the competition layer can obtain the subclassification result through learning, and the linear layer classifies the subclassification result to obtain target classification result [10]. The learning rules of the LVQ neural network combine the mentor learning rules and the competitive learning rules. First, the LVQ neural network is trained on a set of training samples with mentor signals [11]. Usually, each neuron in the competition layer is assigned to an output neuron, and the corresponding weight is generally set to 1, and then a weight matrix of the output layer can be obtained. The columns of the weight matrix are represented as categories, and the rows are represented as subcategories. Generally, the weight matrix is set in advance during training to specify the type of output neuron. The weight matrix data does not change during the training process, and the network learning is carried out by changing the weight matrix. According to the input sample category and the category of the winning neuron, it can be judged whether the current classification is correct. If the classification is correct, the weight vector of the winning neuron is adjusted to the input vector direction, and the classification error is adjusted in the opposite direction [12, 13].

Although competing networks can perform adaptive classification, there are still many problems to be solved. When the learning rate is too fast, the training speed of the network is very fast, but when the weights are updated and the correct classification is achieved, the weights are prone to shock and extremely unstable. When the learning rate is too slow, the training speed of the network is slow, but once the correct classification is achieved, it is not easy to oscillate. Therefore, it is necessary to make a compromise choice between learning rate and network stability. Second, when the vectors belonging to each category are very close to each other, it will cause the weight vectors of the prototypes to interfere with each other, resulting in the destruction of the classification. Third, when the input vector of the neural network is too far away from the corresponding neuron, the neuron may never be able to win and learn in the competition [14].

### 2.2. LVQ Neural Network Algorithm Process

LVQ neural network is a two-layer network, the number of neurons in the first layer is *S*_1_, and the number of neurons in the second layer is *S*_2_. In this neural network, each neuron in the competition layer will be assigned to a neuron in the output layer [15, 16]. The neurons in the competition layer are subcategories, while those in the output layer are categories. Generally, each category can include several subcategories. Therefore, *S*_1_ is usually greater than the number of *S*_2_.

The difference between the LVQ network and other networks is that the net input of the network is not the inner product of the input vector and the weight vector but the direct distance between the input vector and the weight vector [17, 18]. The competition layer of the LVQ neural network calculates which neuron the input vector is closest to, sets the output of this neuron to 1, and sets the output of the rest of the neurons to 0 to obtain the subcategories of the input vector. Then through the calculation of the second layer network, it determines to which class this subclass belongs, to finally determine the class of the input vector. The advantage of this calculation method is that the input vector does not need to be normalized, which simplifies the calculation process.

The net input *n* of the LVQ network is shown in the following formula:

(1) $$\begin{array}{c} \;X_{i}^{1}=-\left\|x_{i}^{1}-p\right\|. \end{array}$$

The vector is expressed as

(2) $$\begin{array}{c} \;X_{i}^{1}=-\left(\begin{array}{c} \left\|x_{1}^{1}-p\right\|\\ \left\|x_{2}^{1}-p\right\|\\ \cdots \\ \left\|x_{i}^{1}-p\right\| \end{array}\right). \end{array}$$

The weight *W* of the first competition layer of the LVQ network starts sample training by assigning a set of randomly smaller initial values. After the samples are trained one by one, the weight vector of the competition layer represents the standard pattern vectors of different categories, which can be realized to recognize and classify the input vector. And when a new vector is input, the network can adjust the weight vector that is closest to it in time and still make it get the correct classification. The category of the input vector is determined by the weight *W* of the second linear layer of the LVQ network. The rows of 2*W* represent classes, and the columns of *W* represent subclasses. Usually several subcategories can be combined into one category [19]. Each column of the weight matrix *W*_2_ has one and only one 1, which means that the subcategory of the column belongs to the category set to 1 row. *W*_2_ means as shown in the following formula:

(3) $$\begin{array}{c} \;W_{ij}^{2}=1⟶\mathrm{indicates}\;\mathrm{that}\;\mathrm{subclass}\;j\;\mathrm{is}\;a\;\mathrm{part}\;\mathrm{of}\;i. \end{array}$$

The basic idea of the LVQ neural network algorithm is to first calculate the neuron of the competitive layer closest to the input vector and find the neuron of the linear output layer connected to it and secondly consider whether the type of the input vector is consistent with the type corresponding to the neuron in the linear output layer. If they are consistent, the weights of the corresponding competing layer neurons are moved along the direction of the input vector; if they are inconsistent, they move in the opposite direction [20]. Specific steps are as follows:

*Step 1.* Initializing the network: initialize the weight vector  *W*_*ij*_^2^ and the learning efficiency  *δ* between the neurons in the input layer and the competition layer.
*Step 2.* Importing the input layer vector: after inputting the initial vector, calculate the distance *di* between the neurons in the competition layer and the input vector according to the following formula:
  (4) $$\begin{array}{c} \;d_{i}=-\left\|X-W_{i}\right\|=\;\underset{n⟶\infty }{\lim}\sqrt{\sum_{j=1}^{n}{\left[X_{j}-W_{ij}\right]}^{2}}, \end{array}$$
where *X* is the input vector and *w*_*ij*_ is the weight between the input layer *j* neuron and the competing layer *i* neuron.
*Step 3*. Determining the winning neuron: find the competitive neuron with the smallest distance from the input vector, determine the winning neuron *k*, set the *k*-th element of the output vector a1 of the competitive layer to 1, and set the rest to 0.
*Step 4*. Calculating the output vector of the linear layer: calculate the value of the output vector of the linear layer and obtain the classification.
*Step 5*. Adjusting the weight: compare the target output with the actual output of the network; if the classification is correct, adjust the direction of the eye input vector; if not, adjust the direction in the reverse direction.
*Step 6*. Updating the learning rate: update the learning efficiency according to the following formula:
  (5) $$\begin{array}{c} \;\delta \left(x\right)=\frac{\delta \left(0\right)\left(x_{j}-x\right)}{x_{j}}. \end{array}$$
*Step 7*. Judgment result: when  *x* < *x*_*j*_,  *k*=*k*+1, return to Step 2 and enter the next sample, repeat the above process, and adjust the weight until  *x*=*x*_*j*_.

During network training, it may appear that the input feature vector is too far away from the neuron, causing the neuron to never win the competition [21–23]. The fraud identification process in accounting based on LVQ neural network is shown in Figure 3.

## 3. Sample Selection and Fraud Risk Identification Index Screening

### 3.1. Sample Selection

Due to the lag in the detection of corporate fraud, fraud is often discovered after the annual fraudulent accounting statements are released. This article is based on the China Securities Regulatory Commission, the website of the Shanghai Stock Exchange and the Shenzhen Stock Exchange. The website publicly disclosed the company violation announcements combined with the listed company violation processing database to determine the fraud samples. Therefore, the sample of this article selects 500 companies that have committed fraudulent activities during the five years from 2015 to 2019 as the fraud samples.

The empirical research sample in this paper includes fraudulent companies and matching companies that are matched with fraudulent companies one-to-one. Therefore, the sample data include 550 companies. The matching sample company is determined according to the Beasley principle. There are 4 specific criteria, namely: (1) the matching company searched for has no fraud in the fraud year of its corresponding fraud company; (2) the asset scale of the matching company and the corresponding fraud company in the previous year is very close, and the difference is less than 30%. (3) the matching company and its corresponding fraud company should be in the same industry and have the same or similar main business; and (4) the matching company and its matching fraud company should be in the same stock exchange market. When the above 4 criteria cannot be met at the same time, the priority shall be given to (2) and (3) provided that (1) must be met.

### 3.2. Screening of Fraud Risk Identification Index

The most critical link in constructing a fraud risk identification model is the selection of fraud risk identification indicators. Indicators with a good identification effect can play a role in accurately predicting and controlling corporate fraud in advance. However, if the indicators are not selected properly, even if the fraud risk identification model is constructed very well, the identification effect is not ideal. This article is based on the fraud triangle theory and selects indicators based on the following three criteria: (1) the selected literature review in this article: in each literature, several indicators have the best results in judging fraud; (2) in view of the difficulty of index data collection and processing, eliminate the indexes that are too complicated and unavailable in the processing process; and (3) important fraud risk identification indicators that have appeared in classic fraud cases: in the literature review part, this article has sorted out the indicators used by a large number of domestic and foreign scholars in the identification of management fraud and screened them in accordance with the above three principles. A total of 11 variables with good discriminating effects were selected and 48 indicators were divided into two pieces of indicators, accounting and nonaccounting indicators. Accounting indicators include six subcategories of profitability, solvency, operating capability, development capability, per share indicators, and asset quality; nonaccounting indicators include five subcategories of equity structure, corporate governance, special transactions and events, audit relationships, and operating pressures. Classification basically covers high-frequency indicators for fraud identification.

## 4. Experimental Results of Combined Neural Network Model

### 4.1. Descriptive Statistics of LVQ Neural Network and Determination of Final Indicators

In order to verify the comprehensiveness and significance of the initially selected index system and to improve the recognition accuracy and efficiency of the fraud risk identification model, this paper will conduct a paired sample *T* test for all the initially determined indicators and conduct a nonparametric Mann–Whitney test. The relevant inspection process is carried out in SPSS17.0. Among them, the qualitative indicators are represented by 1 and 0, mainly including *X*_9_ chairman change, where 1 means change and 0 means no change; *X*_10_ two-time part-time, where part-time is 1, if it is 0; *X*_11_ audit opinion type, where 1 is issued standard audit opinion and 0 means a nonstandard audit opinion issued; *X*_12_ change of the accounting firm, where 1 means change of the accounting firm and 0 means no change of the accounting firm; *X*_12_ avoid ST; that is, whether there are consecutive losses in the previous two years of fraud, where 1 means loss, and 0 indicates that there is no continuous loss.

In order to facilitate data processing and improve the fraud identification effect of the neural network model, this paper sets the fraud company type to 1 and the matching sample company type to 0. Based on pairs of sample data, the 30 accounting indicators and 18 nonaccounting indicators in the abovementioned initially constructed indicator system are tested for significance, and the variables that pass the significance test are selected. Determine the final fraud risk identification indicators. The final identified fraud risk identification indicators and descriptive statistical results are shown in Table 1 and Figures 4 and 5.

The original data have undergone Mann–Whitney rank test and *T* test, and the results show *X*_1_ indicator, *X*5 earnings per share before interest and tax, *X*_7_ two-time concurrent job, *X*_6_ management shareholding ratio, and *X*_10_ audit opinion type. The 3 indicators of ST are significant at the 1% level. The three indicators of *X*_3_ cash flow ratio and *X*_4_ total profit growth rate are significant at the 5% level. The four indicators of *X*_5_ inventory turnover rate, *X*_6_ board of supervisors' shareholding ratio, *X*_7_ state-owned shares ratio, and *X*_8_ other receivables/total assets are significant at the 10% level.  Table 2 and Figure 6 show the descriptive statistics.

### 4.2. Fraud Recognition Effect Test of Combined Neural Network Model

The fraud recognition effect test of the combined neural network model is still completed using the neural network toolbox that comes with MATLAB. The collected 506 pairs of research samples from 2015 to 2019 are divided into two parts, including 326 pairs of training samples and 180 pairs of test sample [18]. Since the recognition rate of the training sample represents the learning effect of the neural network model and cannot explain the fraud recognition effect of the model, the recognition accuracy rate of the test sample is used for comparative analysis. The specific training and test results are shown in Table 3 and Figure 7.

Among the 150 fraud samples, the combined model identified 136 fraudulent companies and misjudged 14 as nonfraud companies. The identification accuracy of fraudulent companies was 88.54%; among 150 matching companies, the LVQ model identified 132 nonfraud companies, 18 were misjudged as fraudulent companies, and the recognition rate of matching companies was 91.54%. From the overall recognition results of fraud companies, the overall fraud recognition rate of the combined neural network model based on LVQ is 90.48%, and the recognition effect is significantly better than any single neural network model (the overall recognition rate of the neural network model based on LVQ is 86.52%, and the overall recognition rate of the neural network model is 93%). Because the training samples and test samples used for the three neural network models are the same, the fraud recognition rate of the three models is comparable.

### 4.3. Robustness Test of Combined Neural Network Model

In order to test whether the recognition effect of the LVQ-based combined neural network fraud risk identification model is stable, this paper selects 100 companies that have fraudulently occurred in 2019 and 100 matching companies found in one-to-one matching with them as research samples to test the combined model fraud and identify the stability, and the specific robustness test results are shown in Figure 8 and Table 4.

Among the 100 fraudulent sample companies, the combination model identified 85 fraudulent companies and misjudged 15 companies, and the fraudulent company identification rate was 85.17%; among the 100 matching sample companies, the combination model identified 89 matching companies, which was incorrect. 11 companies were awarded and the matching company recognition rate was 90.74%. The overall fraud discrimination rate of the combined model is 84.59%, which is slightly lower than the previous overall fraud recognition rate of 90.54%, but the fluctuation range is not large, and it is still higher than the fraud recognition rate of a single neural network model, indicating the fraud recognition of the combined neural network model. The effect is indeed higher than that of a single model, and the effect of fraud identification is stable, which can be used as a discriminant model for corporate fraud.

## 5. Conclusion

The LVQ neural network combines the ideas of competitive learning with supervised learning algorithms. In the process of network learning, the assignment category of input samples is specified through the tutor signal, thereby overcoming the lack of classification information caused by the use of unsupervised learning algorithms in self-organizing networks weakness. The biggest advantage of LVQ neural network is that it cannot only classify linear input data, but also process multidimensional data containing noise interference. Based on the analysis and comparison of LVQ neural network model structure and advantages and disadvantages, this paper further proposes a fraud risk identification model based on LVQ combined neural network. The neural network model with better recognition effect is used as the main preclassification model, and the LVQ neural network as the postclassification model not only effectively processes the data containing noise, but also makes up for the defects that traditional neural network technology cannot subdivide. The above improves the fraud identification effect of the combined model. The same fraud sample was used to test the fraud recognition effect of the combined neural network model, and the overall fraud recognition rate was 90.51%. The research results show that the combined neural network model with complementary advantages and disadvantages is better than a single neural network model in fraud identification. Selecting fraud sample data in 2019 to test the robustness of the combined neural network model, the results show that the overall fraud recognition rate is 90.54%, which is not much different from the previous overall fraud recognition rate of 90.74%. The combined model's recognition effect is relatively stable. Well, it can be used as one of the optional models for the company's fraud risk identification in the future. The research results of this article broaden the thinking of constructing fraud risk identification models in the future. It is no longer limited to a single fraud identification model. It is possible to combine models with good identification effects or complementary advantages and disadvantages to create a new fraud risk identification model. With the rapid development and continuous progress of artificial intelligence technology, it is expected to construct an intelligent fraud risk identification model in the future. According to the different characteristics of each company, the appropriate fraud index system is automatically selected, and the optimal neural network model is constructed for fraud identification. It is no longer limited to specific types of neural network technology.

## Figures and Tables

**Figure 1:** LVQ neural network structure diagram.

**Figure 2:** Data processing process diagram of LVQ neural network model.

**Figure 3:** Fraud identification process in accounting based on LVQ neural network.

**Figure 4:** Final fraud risk identification Mann–Whitney rank test result.

**Figure 5:** Final fraud risk identification *T* test result.

**Figure 6:** Descriptive statistics results.

**Figure 7:** Discrimination results of neural network model training and test samples based on LVQ.

**Figure 8:** Robustness test results.

**Table 1:** Final fraud risk identification index.

Index selection significance	Index name	Mean value		Mann–Whitney rank test		*T* test	
		Fraud	Pairing	*Z* value	*P* value	*t* value	*P* value
Profitability	*X*1 indicator	355	186	−5.121	≤0.001	−3.931	0.0001
Operating capacity	*X*2 inventory turnover rate	29.73	965.23	−1.181	0.249	−1.731	0.0837
Solvency	*X*3 cash flow ratio	0.098	0.201	4.531	≤0.001	−2.109	0.0357
Development ability	*X*4 total profit	0.013	0.114	−4.274	≤0.001	−2.798	0.0063
Per share index	*X*5 before interest and tax stock income	0.340	0.442	−3.134	0.002	−2.599	0.0096

Corporate	*X*6 shareholding ratio of the board of supervisors	2.121	0.011	−0.242	0.002	−2.574	0.056
	*X*7 two-time part-time	0.645	0.125	−2.542	0.068	−1.541	0.005
	*X*8 management shareholding ratio	0.137	0.091	2.846	0 .004	3.026	0.002

Governance	*X*9 proportion of state-owned shares	0.051	0.037	−2.249	0.248	1.679	0.099

Ownership structure	*X*10 audit opinion type	0.054	0.056	−5.121	0.457	1.548	0.005
	*X*11 change of accounting firm	0.125	0.005	−2.125	0.054	1.513	0.008

Auditor relations	*X*12 other receivables/total assets	0.514	0.012	−2.542	0.045	1.158	0.002
Behavioral characteristics	*X*13 avoid ST	0.154	0.005	−1.242	0.002	1.187	0.015

**Table 2:** Descriptive statistics.

Index name	Mean value	Standard deviation	Analysis *N*
*X*_1_ index	0.005	0.055	550
*X*_2_ inventory turnover rate	0.293	0.142	550
*X*_3_ cash flow ratio	0.455	0.006	550
*X*_4_ total cash debt ratio	0.365	0.275	550
*X*_5_ total profit growth rate	0.155	0.133	550
*X*_6_ earnings per share before interest and tax	0.545	0.124	550
*X*_7_ shareholding ratio of the board of supervisors	0.159	0.152	550
*X*_8_ management shareholding ratio	0.086	0.055	550
*X*_9_ proportion of state-owned shares	0.061	0.175	550
*X*_10_ other receivables/total assets	0.078	0.165	550

**Table 3:** Discrimination results of neural network model training and test samples based on LVQ.

Company type	Training samples (320 pairs in total)			Test samples (150 pairs in total)		
	Fraud company	Matching company	Classification accuracy	Fraud company	Matching company	Classification accuracy
Fraud company	305	15	95.45	136	14	88.54
Matching company	18	312	35.98	18	132	91.54
Overall correct rate	93.54			90.48		

**Table 4:** Robustness test.

	Test samples (150 pairs in total)		
	Fraud company	Matching company	Classification accuracy
Fraud company	85	15	85.17
Matching company	11	89	90.74
Overall correct rate	84.59		

## Data Availability

The data used to support the findings of this study are available from the corresponding author upon request.
